The article "Identification of CeRNA Regulatory Networks in Atrial Fibrillation Using Nanodelivery" was published in 2022. Journal: Evid Based Complement Alternat Med.

# Identification of CeRNA Regulatory Networks in Atrial Fibrillation Using Nanodelivery

**DOI:** 10.1155/2022/1046905

**Published:** 2022-09-29

**Authors:** Ping Lin, Lingqiang Meng, Lei Lyu

**Affiliations:** ^1^Department of Cardiology, Dongying Traditional Chinese Medicine Hospital, Dongying 257055, Shandong, China; ^2^Department of Laboratory, Dongying Traditional Chinese Medicine Hospital, Dongying 257055, Shandong, China; ^3^Department of Geriatrics, Dongying Traditional Chinese Medicine Hospital, Dongying 257055, Shandong, China

## Abstract

The initiation and maintenance of AF is a complex biological process that is the ultimate manifestation of many cardiovascular diseases. And the pathogenesis of atrial fibrillation (AF) is unclear. Therefore, this study aimed to find the potential competing endogenous RNAs (ceRNAs) network and molecular dysregulation mechanism associated with AF. GSE135445, GSE2240, and GSE68475 were obtained from the Gene Expression Omnibus (GEO). Differential analysis was utilized to identify the differentially expressed mRNAs, miRNAs, and lncRNAs between AF and sinus rhythms (SR). AF-associated mRNAs and nanomaterials were screened and their biological functions and KEGG signaling pathways were identified. Nanomaterials for targeted delivery are uniquely capable of localizing the delivery of therapeutics and diagnostics to diseased tissues. The target mRNAs and target lncRNAs of differentially expressed miRNAs were identified using TargetScan and LncBase databases. Finally, we constructed the ceRNAs network and its potential molecular regulatory mechanism. We obtained 643 AF-associated mRNAs. They were significantly involved in focal adhesion and the PI3K-Akt signaling pathway. Among the 16 differentially expressed miRNAs identified, 31 differentially expressed target mRNAs, as well as 5 differentially expressed target lncRNAs were identified. Among them, we obtained 2 ceRNAs networks (hsa-miR-125a-5p and hsa-let-7a-3p). The aberrant expression of network target genes in AF mainly activated the HIF-1 signaling pathway. We speculated that the interaction pairs of miR-125a-5p and let-7a-3p with target mRNAs and target lncRNAs may be involved in AF. Our findings have a positive influence on investigating the pathogenesis of AF and identifying potential therapeutic targets.

## 1. Introduction

Atrial fibrillation (AF) is one of the most common arrhythmias and is strongly associated with poor quality of life, stroke, heart failure, and increased mortality [1]. AF has an incidence of up to 4% in modern Western populations and 0.5%–2% in Asian populations [2]. The lifetime risk for people aged 40 to 55 years has been estimated to be between 22% and 26% [3]. In 2010, the estimated number of people living with AF around the world was around 33.5 million [4]. Currently available treatments for AF have limited efficacy, and the mechanisms of development are poorly defined [5, 6]. Therefore, elucidating the exact molecular mechanisms of AF is urgently needed to identify suitable therapeutic targets. AF is one of the final manifestations of diverse disease pathological processes, and its occurrence and maintenance cannot be explained by a single mechanism. Electrophysiological remodeling and structural remodeling have been reported to characterize the pathomechanism of AF [7]. Multiple molecular factors are involved in the progression of AF pathophysiology, including fibrosis, Ca2+ abnormalities, immune-inflammatory responses, and so on [8, 9].

The article "Identification of CeRNA Regulatory Networks in Atrial Fibrillation Using Nanodelivery" was published in 2022. Journal: Evid Based Complement Alternat Med.

Long noncoding RNAs (lncRNAs) are a class of transcripts greater than 200 NT in length that are involved in a variety of biological processes. Dysregulation of lncRNAs was found to be associated with many cardiac diseases, including AF [10]. MicroRNAs (miRNAs) are a class of small noncoding RNAs approximately 18–25 nucleotides in length that negatively regulate the expression of target genes by binding to complementary sequences in 3′-untranslated regions (3′-UTRs) of target mRNAs, thereby promoting their degradation or inhibiting their translation [11]. Therefore, it is important to determine their role in the development of AF and whether they can be used to treat AF. It is well known that lncRNAs can play a certain role as a kind of competing endogenous RNA (ceRNA), thereby sequestering miRNAs away from target mRNAs [12]. These are also the ceRNA regulation guidelines. Bioinformatics analysis provided a new perspective to study the ceRNA involved in AF and laid a foundation for further investigation of their potential roles in AF. The enrichment results of differentially expressed mRNAs were the underlying molecular dysregulation mechanism of AF. Focal adhesion and extracellular matrix (ECM)-receptor interaction were reported to be associated with AF [13]. Focal adhesion group proteins are considered novel disease candidates with the potential to contribute to arrhythmia [14]. Abnormal deposition of ECM, which affects the maintenance of myocardial tissue structure, contributes to the pathological remodeling of AF [15]. There is evidence that downregulation of PI3K-Akt expression is associated with an increased incidence of AF in diabetic rats [16]. The PI3K-Akt pathway was confirmed to reduce the incidence of AF and attenuate atrial fibrosis [17].

Therefore, we aimed to screen differential genes in patients with AF, identify networks of AF-related molecular biological mechanisms, and explore key regulators during the progression of AF. In this study, the ceRNA network was established to facilitate the search for diagnostic and therapeutic targets associated with AF. In addition, enrichment analysis was performed on the differentially expressed mRNAs, and the signaling pathways regulated by the ceRNA network were identified. Several molecular mechanisms involved in cardiovascular remodeling are further highlighted. We believe that hsa-miR-125a-5p, hsa-let-7a-3p, and target genes may participate in the pathogenesis of AF through the HIF-1 signaling pathway.

The article "Identification of CeRNA Regulatory Networks in Atrial Fibrillation Using Nanodelivery" was published in 2022. Journal: Evid Based Complement Alternat Med.

## 2. Materials and Methods

### 2.1. Data Collection

GSE135445 included mRNA and lncRNA expression profiles of epicardial adipose samples from patients with persistent nonvalvular AF (*n* = 6) and sinus rhythm (SR, *n* = 6) based on the GPL20301 platform. GSE2240 included an mRNA expression profile of atrial tissue from 10 permanent AF and 20 SR based on the GPL97 platform. GSE68475 included miRNA expression profile of atrial right appendages from 10 samples were from patients with persistent AF and 11 normal SR based on the GPL15018 platform.

### 2.2. Difference Analysis

Difference analysis for mRNAs and lncRNAs between AF and SR in GSE135445 was performed using the edger R package [18]. The limma R package [19] was used for the difference analysis of mRNAs and miRNAs between AF and SR in GSE2240 and GSE68475. *P* value < 0.05 was used to define significant differentially expressed mRNAs (DEmRs), differentially expressed lncRNAs (DElncRs), and differentially expressed miRNAs (DEmiRs) in the results of the difference analysis.

### 2.3. Functional and Pathway Enrichment

The enrichment analysis of Gene Ontology (GO) and Kyoto Encyclopedia of Genes and Genomes (KEGG) pathway enrichment analysis for mRNAs was performed using the clusterProfiler R package [20]. The biological process (BP) was one kind of GO enrichment. The *P* < 0.05 was set as the threshold of statistical significance. Gene set variation analysis (GSVA) was performed using the GSVA R package to display enrichment results of target mRNAs. To identify the underlying molecular dysregulation mechanisms of AF, we performed an enrichment analysis of AF-associated mRNAs. These mRNAs were enriched to three ontologies of GO: cellular component (CC), molecular function (MF), and biological process (BP).

### 2.4. Immune Cell Infiltration

The xCell R package [21] was used to assign and visualize 31 types of immune cells in AF and SR samples based on ssGSEA (single-sample gene set enrichment analysis) in GSVA (gene set variation analysis). *P* value <0.05 was considered statistically significant for xCell scores between AF and SR which were calculated with the limma R package.

The article "Identification of CeRNA Regulatory Networks in Atrial Fibrillation Using Nanodelivery" was published in 2022. Journal: Evid Based Complement Alternat Med.

### 2.5. Target Prediction and CeRNA Network Construction

The LncBase Predicted v.2 was used to predict the target lncRNAs regulated by differentially expressed miRNAs. The screening threshold was set as 0.7. Then, the target mRNAs regulated by differentially expressed miRNAs were predicted using TargetScan (https://www.targetscan.org/vert_72/) database. The ceRNA network was established from the differentially expressed lncRNAs, miRNAs, and mRNAs. CeRNA networks identified by us included a downregulated lncRNA (AC125807.2) that was regulated by upregulated hsa-miR-125a-5p, as well as downregulated mRNAs (EGFR, MACF1, TRPS1, EEF1A1, MASP1, PANX1, PUM2, CGNL1, NPM1, and TFRC). Upregulated lncRNA (LINC01139) and upregulated mRNA (SRI) were regulated by downregulated hsa-let-7a-3p.

## 3. Results

### 3.1. Identification of AF-Associated mRNAs

To identify AF-associated mRNAs, we performed differential expression analysis of mRNAs in GSE135445. By threshold screening, we obtained 1556 differentially expressed mRNAs between AF and SR (Figure 1(a)). These included 733 upregulated differentially expressed and 823 downregulated differentially expressed (Figure 1(b)). We obtained 7084 differentially expressed mRNAs in GSE2240, and by comparing them with those of GSE135445, we identified 643 common differentially expressed mRNAs (Figure 1(c)). There were significant differences in the expression of common mRNAs between AF and SR samples in GSE2240 (Figure 1(d)), and they may be AF-associated mRNAs.

### 3.2. Biological Functions of Common mRNAs

Figure 2(a) shows the top 10 GO terms in AF-associated mRNAs enrichment. In CC results, we identified significantly enriched focal adhesion, cytoskeleton, and secretory granule lumen. RNA binding, cadherin binding, and protein kinase binding were significantly enriched in MF. And regulation of cell migration, regulation of angiogenesis, and neutrophil-mediated immunity were significantly enriched in BP. In addition, we found focal adhesion, PI3K-Akt signaling pathway, and ECM-receptor interaction to be significantly enriched in KEGG results (Figure 2(b)). On the other hand, we calculated the infiltration of immune cells in AF patients. CD8+ naïve T cell and Th1 cell infiltration were significantly higher in AF, whereas macrophage M1 and Th2 cell infiltration were significantly lower in AF, compared with SR (Figure 2(c)).

### 3.3. Differentially Expressed MiRNAs and lncRNAs

Sixteen differentially expressed miRNAs in GSE68475 were identified in AF patients after comparison with Sr (Figure 3(a)). In GSE135445, we found 286 differentially expressed lncRNAs between AF and SR (Figure 3(b)). Using the TargetScan database, we identified 529 target mRNAs of the differentially expressed miRNAs. Comparing with the differentially expressed mRNAs, we obtained 31 differentially expressed target mRNAs (Figure 3(c)). Using the LncBase database, we identified 2358 target lncRNAs of differentially expressed miRNAs. Compared with the differentially expressed lncRNAs, we obtained 5 differentially expressed target lncRNAs (Figure 3(c)).

The article "Identification of CeRNA Regulatory Networks in Atrial Fibrillation Using Nanodelivery" was published in 2022. Journal: Evid Based Complement Alternat Med.

### 3.4. CeRNA (DElncRs-DEmiRs-DEmRs) Regulatory Network

According to the ceRNA regulation guidelines, the two ceRNA networks were established by Cytoscape software (Figure 4(a)), which included upregulated hsa-miR-125a-5p, downregulated lncRNAs, and mRNAs target, as well as downregulated hsa-let-7a-3p, upregulated lncRNAs, and mRNAs target. The results of enrichment analysis showed that the target mRNAs were mainly involved in the HIF-1 signaling pathway, endocytosis, and ferroptosis (Figure 4(b)). Using GSVA, we evaluated the expression of these signaling pathways in AF patients (Figure 4(c)). Comparison with SR found that the GnRH signaling pathway was inhibited in AF and the other signaling pathways were all activated in AF (Figure 4(d)):

## 4. Discussion

In recent years, with the rapid development of high-throughput technologies, researchers have been able to observe changes in molecular regulatory mechanisms at the gene expression level. In this study, we used transcriptome data of AF patients from public databases containing mRNAs, lncRNAs, and miRNAs. A total of 643 differentially expressed mRNAs, 286 differentially expressed lncRNAs, and 16 differentially expressed miRNAs were identified. In the results of enrichment analysis, the differentially expressed mRNAs were mainly associated with focal adhesion, PI3K-Akt signaling pathway, and ECM-receptor interaction. In addition, we identified a significant infiltration level of immune cells in AF. Importantly, we successfully constructed a ceRNA network to further understand the underlying regulatory mechanism of AF.

Interestingly, we identified 2 ceRNA networks. Consistent with the results of our analysis, miR-125a-5p was upregulated in patients with AF [22]. Studies have shown that genetic polymorphisms of miR-125a are associated with the recurrence of AF [23]. Moreover, dysregulated miR-125a-5p expression is associated with the formation of vascular plaques and vascular restenosis [24]. In addition, hsa-let-7a-3p expression was downregulated in AF compared with SR [25]. Khudiakov et al. showed that hsa-let-7a-3p was abnormally expressed in cardiovascular disease [26]. It is shown that let-7a-3p acts as a tumor suppressor and participates in the regulatory processes of proliferation and apoptosis in cancer cells [27].

The article "Identification of CeRNA Regulatory Networks in Atrial Fibrillation Using Nanodelivery" was published in 2022. Journal: Evid Based Complement Alternat Med.

Here, the results of our analysis suggest that AC125807.2 is a regulator of AF and competitively binds to miR-125a-5p with multiple target mRNAs. Among them, p38-mitogen-activated protein kinase has been implicated in AF and atrial remodeling after epidermal growth factor receptor (EGFR) activation [28]. EGFR is required for cardiovascular function and its deletion produces cardiac damaging effects [29]. MACF1 has a regulatory effect on the focal adhesion of the cytoskeleton [30]. In addition, LINC01139 is competitively bound to let-7a-3p with SRI, thereby participating in the molecular regulation of AF. Sorcin (SRI), an accessory binding protein, regulates sarcoplasmic reticulum Ca2+ release and has important functions in the pathogenesis of AF [31, 32]. Seidler et al. showed that SRI overexpression affects cardiomyocyte excitation-contraction coupling [33].

Among the signaling pathways regulated by the ceRNA network, we found that the HIF-1 signaling pathway was significantly activated in AF. Hypoxia-induciblefactor-1 (HIF-1) is a regulator that regulates the body's response to hypoxia-induced angiogenesis [34]. Atrial hypoxia promotes atrial fibrillation substrate formation by promoting atrial structural remodeling [35]. In the early response of cardiomyocytes to AF, the expression of genes of HIF-1*α* was increased in synchrony with the onset of atrial myelofibrosis [36]. Activation of the gonadotropin-releasing hormone (GnRH) receptor is associated with coronary heart disease and myocardial infarction [37]. However, in the results of our analysis, the GnRH signaling pathway was significantly inhibited. This is consistent with the findings of Chiang et al. [38]. These results suggest that the ceRNA network may be involved in the development of AF through the regulatory mechanisms of HIF-1 and GnRH signaling during the pathogenesis of AF, but these mechanisms require further investigation.

## 5. Conclusion

We identified two ceRNA networks, including hsa-miR-125a-5p, hsa-let-7a-3p, and target genes. They may participate in the pathogenesis of AF through the HIF-1 signaling pathway. These results provide a partial description of the comprehensive regulatory network of AF, which may help provide new insights into the pathogenesis of AF and identify potential therapeutic targets. However, there are also certain limitations in this study. First, considering our low number of analyzed samples, more samples are needed. Second, we provided two sets of AF-related ceRNA networks, but further experimental validation is needed. We hope to conduct further studies in large-scale clinical samples to identify potential regulatory mechanistic memory therapeutic targets.

The article "Identification of CeRNA Regulatory Networks in Atrial Fibrillation Using Nanodelivery" was published in 2022. Journal: Evid Based Complement Alternat Med.

## Figures and Tables

**Figure 1:** Screening of differentially expressed mRNAs between AF and SR. (a). Heatmap of differentially expressed mRNAs between AF and SR in GSE135445. (b). Volcano plot of differentially expressed mRNAs between AF and SR in GSE135445. Red is upregulated and blue is downregulated. (c). Venn diagram of differentially expressed mRNAs in GSE135445 and GSE2240. (d). Heatmap of common mRNAs in GSE2240.

**Figure 2:** Identification of potential molecular maladjustment mechanisms of AF. (a). The top 10 GO terms in AF associated mRNAs enrichment. (b). Significantly enriched KEGG pathways of AF-associated mRNAs. (c). Levels of immune cell infiltration in patients with AF and SR. ^*∗*^*P* < 0.05, ^*∗∗*^*P* < 0.01, ^*∗∗∗*^*P* < 0.001.

**Figure 3:** Identification of differentially expressed miRNAs and prediction of their target lncRNAs and mRNAs. (a). The differentially expressed miRNAs between AF and SR in GSE68475. (b). The differentially expressed lncRNAs between AF and SR in GSE135445. (c). The intersection of target mRNAs and differentially expressed mRNAs. (d). The intersection of target lncRNAs and differentially expressed lncRNAs.

**Figure 4:** The lncRNA-miRNA-mRNA network in AF. (a). The ceRNA network in AF. Rectangles, triangles, and circles represent lncRNAs, miRNAs, and mRNAs, respectively. (b). Significant KEGG signaling pathways are involved in the target genes. (c). Heatmap of the score of signaling pathways calculated GSVA in AF and SR. (d). Differential analysis identified signaling pathways activated or inhibited in AF compared with SR.

## Data Availability

The datasets used and/or analyzed during the current study are available from the corresponding author upon reasonable request.
